This article has been retracted.

# microRNA-324-3p suppresses the aggressive ovarian cancer by targeting *WNK2*/RAS pathway

**DOI:** 10.1080/21655979.2022.2056314

**Published:** 2022-05-13

**Authors:** Fengjie Li, Zhen Liang, Yongqin Jia, Panyang Zhang, Kaijian Ling, Yanzhou Wang, Zhiqing Liang

**Affiliations:** a Department of Obstetrics and Gynecology, Southwest Hospital, Third Military Medical University, Chongqing, Sichuan , China; b Department of Plastic and Reconstructive Surgery, Xijing Hospital, Fourth Military Medical University, Xi’an, Shaanxi, China

**Keywords:** Ovarian cancer, microRNA, WNK2, miR-324-3p, proliferation and invasion, RAS pathway

## Abstract

Ovarian cancer (OC) has the highest mortality rate among gynecological cancers, which progresses owing to dysregulated microRNAs (miRNAs) expression. Our study attempts to reveal the mechanism by which decreased miR-324-3p expression suppresses OC proliferation. Quantitative real-time PCR, western blotting, in situ hybridization, and immunohistochemistry were performed to estimate miR-324-3p and WNK2 expression levels in OC cells and tissues. Cell Counting Kit-8, colony formation, EdU, and transwell assays were performed to analyze the influence of miR-324-3p and WNK2 on the proliferation and invasion ability of OC cells. Subsequently, xenograft models were established to examine the effects of WNK2 on OC cell proliferation in vivo, and databases and luciferase reporter assays were used to test the relationship between miR-324-3p and *WNK2* expression. Then, we showed that miR-324-3p expression is decreased in OC cells and tissues, indicating its inhibitory effect on OC cell proliferation. Quantitative real-time PCR and luciferase reporter assays demonstrated that miR-324-3p inhibited *WNK2* expression by directly binding to its 3’ untranslated region. WNK2, an upregulated kinase, promotes the proliferation and invasion of OC cells by activating the RAS pathway. Moreover, WNK2 can partly reverse the inhibitory effects of miR-324-3p on OC cell proliferation. Hence, we demonstrate that miR-324-3p suppressed ovarian cancer progression by targeting the *WNK2*/RAS pathway. Our study provides theoretical evidence for the clinical application potential of miR-324-3p.

## Highlights

• WNK2 induces ovarian cancer cell proliferation and its invasion ability.
• Mechanism of ovarian cancer inhibition by miR-324-3p is revealed.
• miR-324-3p inhibits OC proliferation by binding to 3’ untranslated region of WNK2
• Suppressive role of miR-324-3p in ovarian cancer relies on WNK2-RAS pathway.
• WNK2 facilitates ovarian cancer progression by activating the RAS pathway.

## 1. Introduction

Ovarian cancer (OC) has the highest mortality rate among gynecological cancers types. In 2020, 313959 women were diagnosed with OC, of which 207252 of them died [1,2]. Primary cytoreductive surgery followed by chemotherapy is the commonly used treatment for OC [3]. Despite continuous development in surgical skills and chemotherapy techniques, the 5-year survival rate of OC remains below 40% [4]. Unveiling OC progression mechanism and developing new therapeutic targets is crucial for improving patient outcomes.

Genomic alterations are the hallmarks of OC, and 98% of the altered genomes are non-coding genes [5–7]. MicroRNAs (miRNAs) are important non-coding RNAs of the non-coding genome and are 19–25 nucleotides long. They degrade mRNAs by binding complementarily to the target mRNAs [8,9]. In addition, miRNAs play vital roles in regulating several processes in tumor progression, including proliferation, metastasis, and invasion [10,11]. Furthermore, miR-324-3p is abnormally expressed in tumors, which plays critical roles in regulating of the malignant phenotypes of various cancer cells. For instance, miR-324-3p overexpression promotes the proliferation of hepatocellular cancer cells [12]. In pancreatic, breast, and nasopharyngeal cancers, it acted as a tumor suppressor by targeting oncogenes such as *ACK1,TGF-β1* and *WNT2B* [13–15]. The PI3K/AKT, MAPK and Wnt/β-catenin pathways are the downstream effectors of miR-324-3p [16–18]. Moreover, miR-324-3p can be used as a prognostic signature for childhood acute lymphoblastic leukemia, lung, bladder, liver, colorectal, and pancreatic cancers [19–24]. Furthermore, decreased miR-324-3p expression inhibits OC development [25]. However, the underlying mechanism has not yet been elucidated.

WNK2 is a member of WNK kinase family [26]. It is a cytoplasmic protein located on chromosome 9q22.31. It has multiple domains and a molecular weight of 243 kDa. WNK2 was first found to play a vital role in ion transport [27]. However, in recent years, its vital role in cancer development attracted considerable attention. To date, WNK2 acts as a tumor suppressor in gliomas and hepatocellular, gastric, breast, colon cancers [28–31]. For example, WNK2 suppresses cervical cancer by negatively modulating the MEK1/ERK1/2 pathway [32]. Moreover, growing evidences show that some vital miRNAs and lncRNAs regulate tumorigenesis by targeting *WNK2*. For instance, miRNA-370 promotes breast cancer development by suppressing *WNK2*, and LINC00858 enhances gastric cancer proliferation by reducing *WNK2* promoter methylation [30,33]. However, the role, clinical significance, and molecular mechanisms of WNK2 in ovarian carcinogenesis remain unclear.

This study aimed to verify the function and explore the mechanism of miR-324-3p in OC progression. Bioinformatics websites predicted that miR-324-3p targets *WNK2*. To the best of our knowledge, our study is one of the first to reveal the underlying mechanism by which miR-324-3p inhibits OC, and the first to reveal the tumor promoting roles of WNK2 in OC. By elucidating how miR-324-3p and WNK2 regulate the malignant behaviors of OC, we provided the theoretical foundations for the clinical application of miR-324-3p.

## 2. Materials and methods

### 2.1 In situ hybridization

Tissue microarray HOvaC070PT01, containing 70 OC samples and adjacent normal epithelial tissues samples, was purchased from Shanghai Outdo Biotech Co., Ltd. (Shanghai, China). An in situ hybridization kit (Boster, Bio, CA, USA) was used in detecting miR-324-3p expression, which included phosphate buffered saline (PBS) buffer, 2x saline sodium citrate (SSC), 4% formalin with 1/1000 diethylpyrocarbonate (DEPC), 10x pepsin, prehybridization solution, and miR-324-3p probe hybridization solution. In addition, nonspecific antigen-blocking, biotinylated mouse antidigoxin, streptavidin–biotin complex peroxidase (SABC-POD), and biotinylated peroxidase were included in the kit. The sequence of the miR-324-3p probe was 5’-CCA GCA GCA CCT GGG GCA GTG GG-3’. First, methanol and 30% H_2_O_2_ (50:1) were added to the microarray and incubated for 30 min. After washing three times with distilled water, 3% citric acid with pepsin was dripped onto the microarray to expose the nucleic acid fragments. Subsequently, pepsin was successively washed with PBS and distilled water. Then, 4% formalin was used to fix the microarrays. The microarray was then placed in an incubator (37°C) for 2 h with a pre-hybridization solution, and the probe was hybridized overnight at 37°C. The next day, the microarray was washed with preheated 2x SSC, 0.5x SSC, and 0.2x SSC (37°C), successively. Biotinylated digoxin was incubated following nonspecific antigen blocking. Finally, SABC incubation, biotinylated peroxidase incubation, diaminobenzene (DAB) staining, dehydration, and neutral resin sealing were processed sequentially [34].

### 2.2 Cell culture

A human ovarian epithelial cell line (IOSE-80) and high-grade serous adenocarcinoma cell lines (CAOV3, A2780, and SKOV3 cells) were purchased from the American Type Culture Collection (ATCC, Manassas, VA, USA). All cell lines were cultured in Dulbecco’s modified Eagle’s medium (DMEM) containing 10% fetal bovine serum (Gibco, Gaithersburg, MD, USA). Subsequently, 100 U/mL of penicillin and 0.1 mg/mL of streptomycin (Beyotime, Shanghai, China) were added to the culture medium. All cell lines were cultured at 37°C in an incubator under a 5% CO_2_ humidified atmosphere.

### 2.3 RNA extraction and quantitative real-time PCR (RT-qPCR)

After 48 h of transfection, RNA was extracted using TRIzol reagent (Takara, Kyoto, Japan). Reverse transcription and RNA detection were performed using HiScript III-RT SuperMix and ChamQ Universal SYBR qPCR Master Mix (MixVazyme, Piscataway, USA). Then, PCR amplification of target genes was conducted as follows: 95°C for 3 min, 95°C for 10s, 57°C for 30s (39 cycles), 65°C for 5 s, and 95°C for 0.5 s. U6 and GAPDH were used in normalizing miR-324-3p or *WNK2* expression, respectively. The primer sequences for the target genes are listed as follows: miR-324-3p primer: CTC AAC TGG TGT CGT GGA GTC GGC AAT TCA GTT GAG CAG CACC; miR-324-3p F: 5’-ACT GCC CCA GGT GCTG-3’ and R: 5’-CTC AAC TGG TGT CGT GGA-3’; U6 F: 5’-CTC GCT TCG GCA GCA CA-3’ and R: 5’-AAC GCT TCA CGA ATT TGC GT-3’; *WNK2* F: 5’-TGG TTC ATC ATC TGT CCG-3’ and R: 5’-AAG CTG GGT TGT TCC TT-3’, and *GAPDH* F: 5’-AGC CAC ATC GCT CAG ACAC-3’ and R: 5’-TTA AAA GCA GCC CTG GTG AC-3’ [34].

### 2.4 Transfection and transduction

The cells were seeded into the plate the day before. Transfection was performed the following day after the cell density reached approximately 70% confluence. Then 50 nM si-RNA, miR-324-3p mimic, mimic NC, miR-324-3p inhibitor, inhibitor NC (Ribobio, Guangzhou, China), or 3000 ng plasmids (Genechem Co., Ltd., Shanghai, China) were added to the medium without serum. After 6 h of transfection, the medium was placed with a fresh medium containing 10% serum. Lipo3.0 (Thermo Fisher, Waltham, USA) was used to increase transfection efficiency. The related sequences are listed as follows: si-WNK2-1: CAAGGACAATGGAGCCATA; si-WNK2-2: GGAGTATGCTAGGCTATGA; and si-WNK2-3: CGATGAAATTGCCACGTAT. We transduced the constructed lentivirus (TsingKe, Beijing, China) into adherent cells (MOI = 30) to establish cell lines with stable *WNK2* knockdown. After 2 μg/mL puromycin screening, the surviving cells were used for subsequent analysis [35].

### 2.5 Cell proliferation assays

3000 pretreated cells were incubated into 96-well plates to examine the effects of miR-324-3p and WNK2 on cancer cells. Cell viability was measured periodically using a cell counting kit (CCK-8) (Beyotime, Shanghai, China). All the experiments were performed in triplicate, and three holes were designed per group. For colony formation assay, 2000 cancer cells (per well) were cultured in 12-well plates. After 2 weeks, the cells were fixed with 4% paraformaldehyde (Boster, CA, USA) and stained with crystal violet (Beyotime, Shanghai, China). Then, Image J software was used to count the colonies [36].

### 2.6 EdU staining assays

EdU assay kits (Beyotime, Shanghai, China) were used to test cell proliferation to further confirm the effect of the target gene on proliferation. After transfection for 48 h, the OC cells were incubated with EdU (50 µm) for 2 h at 37°C, which were then fixed with 4% paraformaldehyde and permeabilized with 0.3% Triton X-100. Next, the cells were incubated with the ready-to-use click reaction mixture in the dark for 30 min. Finally, they were incubated with Hoechst 33342 (1/1000) for 10 min to stain nuclei. Images were captured using a BX53 Olympus fluorescence microscope (Beijing, China).

### 2.7 Dual-luciferase reporter assay

The bioinformatics website TargetScan (http://www.targetscan.org/) predicts the two potential binding sites for WNK2 and miR-324-3p. The wild-type or three mutant WNK2 3'UTR binding site sequences were cloned into pmirGLO luciferase vectors (TsingKe, Beijing, China). Next, 2 × 10^4^293 T cells were plated in a 96-well plate. In the following day, luciferase vectors and miR-324-3p mimics were transfected into the plates. A dual luciferase assay system (Promega, USA) was used after 48 h to measure binding affinity [36].

### 2.8 Cell lysis and western blot

RIPA lysis buffer combined with a 1x cocktail (Beyotime, Shanghai, China) was used to extract proteins. We used protein assay kits (Thermo, Waltham, Massachusetts, USA) to quantify the protein concentration and maintain an equal loading quantity for each sample. For each sample, equal protein amounts were was loaded onto SDS-PAGE gels. After the proteins were transferred onto polyvinylidene fluoride (PVDF) membranes, we blocked the membranes with 5% defatted milk powder at room temperature. The PVDF membranes were then incubated overnight with primary antibodies at 4°C. The primary antibodies used in this study are anti-WNK2 antibody (cat: ab192397, 1:500, Abcam) and anti-actin antibody (cat: ab179467, 1:2000, Abcam). The next day, after the PVDF membranes were washed with Tris-buffered saline containing 0.1% Tween 20 (TBST), they were incubated with the following secondary antibodies: anti-mouse IgG, HRP-linked antibody (cat:7076, 1:5000, CST) and anti-rabbit IgG, HRP-linked antibody (cat:7074, 1:5000, CST). Finally, the band images were captured using a Vilber chemiluminescence image instrument (Shanghai, China) [35].

### 2.9 Immunofluorescence staining

OC cells (SKOV3) were incubated in a 35 mm dish for 24 h before they were fixed with 4% paraformaldehyde. Next, the cells were incubated in 0.1% Triton for another 10 min and were then incubated with the WNK2 antibody (ab239037, 200:1) overnight in the dark. Finally, the images were captured using a Zeiss 880 (Tokyo, Japan).

### 2.10 Immunohistochemistry

The tissue microarray HOvaC160Su01 was purchased from Shanghai Outdo Biotech Co., Ltd (Shanghai, China), which contained 160 OC samples and adjacent normal epithelial tissue samples. HOvaC160Su01 was supplemented with patients’ prognostic information. We performed immunohistochemistry on microarray HOvaC160Su01 to detect WNK2 expression and its clinical significance in OC. The microarrays were then deparaffinized after 4 h of heating in an incubator and immersion in xylene. After antigen retrieval, the microarrays were immersed in 3% H_2_O_2_ to block nonspecific antigens. Then, the primary anti-WNK2 antibody (cat: D262500, 1:200, Sangon Biotech) was incubated on the microarray at 4°C overnight. The following day, 3,3-diaminobenzidine (DAB) staining was performed after secondary antibody incubation. Finally, dehydration and neutral resin sealing were carried out. The immunohistochemistry kit (Gene Tech Company Limited, Shanghai, China) contained nonspecific antigen blockers, antigen retrieval solution, secondary antibodies, and DAB stain. The intensity was quantified by multiplying the staining score of the target gene by the positive area proportion [37].

### 2.11 Transwell assay

The transwell assay was performed to analyze the invasive ability of the cells. Cells (2 × 10^4^) were plated into a upper transwell chamber (Corning, New York, USA) in a serum-free medium. The bottom was immersed in a medium containing 10% serum. An 8 µm pore membrane was in the middle. After 48 h, noninvasive cells were removed from the top layer of the membrane using a cotton swab. Invasive cells were fixed with 4% paraformaldehyde and stained with crystal violet. Finally, images were captured using an Olympus BX53 microscope (Tokyo, Japan) [36].

### 2.12 Xenograft model

Ten 6-week-old female nude mice were purchased from Beijing Huafukang Co., Ltd., (Beijing, China) to evaluate whether WNK2 promoted ovarian cancer progression in vivo. The animals were raised at the Animal Center of Army Medical University. All the experiments were performed in accordance with the rules and regulations of the Animal Ethics Committee of the First Affiliated Hospital, Army Medical University (Third Military Medical University). All invasive surgeries were performed under anesthesia. We randomly divided the mice into two groups: sh-NC and sh-WNK2, with five mice per group. Then, we suspended 1 × 10^6^ stable cells (NC and sh-WNK2) in 50 μL of PBS and 50 μL of Matrigel (Corning, USA) to establish tumor models for each nude mouse. Then, 100 μL of cell suspension was administered into the dorsal flanks of the mice. Given that visible lumps were observed, we measured the tumor size with a caliper twice daily. The tumor volumes were equal to (width^2^  ×  length)/2. The mice were euthanized after three weeks, and the tumors were dissected for further analysis.

### 2.13 Proteome profiling of phosphorylation modification

As a serine or threonine kinase, WNK2 may promote tumor progression by activating these pathways. Thus, we performed a phosphorylation modification proteome study of WNK2 after establishing a WNK2-knockdown stable cell line of SKOV3. Then, we collected the cells and PTM Biolabs, Incorporation conducted the proteome analysis. Proteins and peptides phosphorylated by WNK2 were elucidated through protein extraction, enzyme digestion, modified peptide enrichment, mass spectrum analysis, and bioinformatics analysis.

### 2.14 RAS activity detection

To verify the phosphorylation modification sequencing results, we purchased the RAS activity detection kit from Wuhan New East Biosciences Co., Ltd. (Wuhan, China). We cultured OC cells (sh-NC SKOV3, sh-WNK2 SKOV3, sh-NC CAOV3, and sh-WNK2 CAOV3) in 10 cm dishes. Then, we extracted 1.5 mg of proteins from each sample and incubated them with active RAS antibody and protein A/G beads for 2 h. After washing the beads three times, 20 µL of 2x loading buffer was added and the protein was heated at 100°C for 10 min. Subsequently, western blotting was performed as previously described.

### 2.15 Statistical analysis

Statistical analysis and graphing were conducted using IBM SPSS Statistics 23 or GraphPad Prism 8. Paired t-tests and independent-sample t-tests were used to analyze differences between the groups. Cox regression analysis was used for survival analysis. Pearson’s chi-squared test was used to test the association between clinicopathological parameters and target genes. In all tests, statistical significance was set at *p* < 0.05.

## 3. Results

miRNAs play vital roles in the regulation of tumor progression. Sufficient evidence confirms that OC progression is caused by dysregulated miRNAs. In OC, miR-324-3p suppresses tumor development. However, the role of miR-324-3p in OC remains unclear. In this study, we performed correlation experiments and functional experiments to validate that miR-324-3p suppresses OC by targeting the WNK2/RAS pathway. Our research provides the theoretical evidence for its future clinical application as a potential therapeutic target for OC treatment.

### 3.1 Downregulated miR-324-3p is a tumor suppressor in OC

RNA in situ hybridization was performed to detect the expression of miR-324-3p in adjacent normal epithelial tissues and OC tissues. The results confirmed that miR-324-3p distinctly decreased in OC tissues compared to adjacent ovarian epithelial tissues (*P = 0.041; Figure 1(a,b) and Table 1). RT-qPCR showed that miR-324-3p expression in the OC cells (A2780, CAOV3, and SKOV3) was lower than that in IOSE-80 cells (Figure 1(c)). We successfully overexpressed or inhibited miR-324-3p to determine its role in OC cells. CCK-8, EdU, and colony formation assays showed that the proliferation of A2780 and CAOV3 cells was repressed by miR-324-3p upregulation (Figure 1(d-h)). The decrease in miR-324-3p expression promotes the OC cell proliferation (Figure 1(e-i)).

**Figure 1.** Decreased miR-324-3p plays a tumor suppressive role in OC. (a-b) The levels of miR-324-3p in OC tissues were significantly decreased (*P = 0.041). (c) The expression of miR-324-3p in OC cell lines was evaluated by RT-qPCR. (d) CCK-8 analysis illustrated the effect of miR-324-3p mimics on OC cell viability. (e) the effect of miR-324-3p inhibitors on OC cell viability. (f-g) EdU assay and (h-i) Colony formation assay evaluated the viability of OC cells after transfection of miR-324-3p mimics or inhibitor.

**Table 1.** MiR-324-3p was decreased in ovarian cancer tissues p < 0.05

Parameters	Total (n = 68)		P-value
	High miR-324-3p expression (46)	Low miR-324-3p expression (19)	
			Pathology types
Boderline tumors	5	0	
Serous carcinoma	20	16	0.02*
Mucinous carcinoma	7	0	
germ cell tumor	2	2	0.046*
Other pathology types	12	1	
			Ages (years)
≧55	25	10	0.402
<55	14	9	

### 3.2 miR-324-3p directly targets WNK2

Bioinformatics websites predicted that miR-324-3p targets WNK2. On the TargetScan website (http://www.targetscan.org/), two potential binding sites were identified between 3'UTR of *WNK2* and miR-324-3p (Figure 3(a)). We conducted a luciferase assay to determine whether miR-324-3p directly binds to *WNK2*. The reporter genes *WNK2*-3'WT, *WNK2*-3'UTR-MUT1, *WNK2*-3'UTR-MUT2, and *WNK2*-3'UTR-MUT3 were transfected into 293 T cells. miR-324-3p mimics significantly decreased the luciferase activity of *WNK2*-3'UTR-WT and mutated *WNK2*-3'UTR-MUT1 (*P < 0.05). However, no changes were observed on *WNK2*-3'UTR-MUT2 and *WNK2*-3'UTR-MUT3 (Figure 3(b)), which indicates that miR-324-3p binds to 3'UTR of *WNK2* directly at 941–947 bp. Thus, *WNK2* may be a strong regulatory target of miR-324-3p. Moreover, we transfected miR-324-3p mimics or inhibitors into A2780 and CAOV3 cells to verify whether miR-324-3p regulates WNK2. Then, we found that the mRNA and protein levels of WNK2 decreased when miR-324-3p expression increased in A2780 and CAOV3 cells (Figure 3(c-e)). In contrast, the expression of WNK2 increased when miR-324-3p was inhibited (Figure 3(d-f)). In summary, we provided evidences that miR-324-3p may decrease WNK2 by binding with its 3'UTR.

**Figure 3.** miR-324-3p negatively regulates WNK2 expression in mRNA and protein levels by targeting its’ 3'UTR directly. (a-b) miR-324-3p inhibited the luciferase activities of constructs comprising the wild-type and mutated binding sites (4287–4294) in WNK2 3'UTR. (c-d) mRNA expression of WNK2 was regulated by miR-324-3p. (e-f) Protein changes of WNK2 after miR-324-p was overexpressed or decreased in OC cells. ** P < 0.01, *** P < 0.001.

### 3.3 Expression of WNK2 is negatively correlated with miR-324-3p in OC

RT-qPCR and Western blotting verified WNK2 was significantly upregulated in three OC cell lines (SKOV3, CAOV3, and A2780 cells) at both RNA and protein levels (Figure 2(a,b)). Immunofluorescence analysis showed that WNK2 was localized in the cytoplasm of SKOV3 cells (Figure 2(c)). As shown in the Gene Expression Profiling Interactive Analysis (GEPIA) database, (http://gepia.cancer-pku.cn/) and Human Atlas Protein database (https://www.proteinatlas.org/), WNK2 was overexpressed in the OC tissues compared to normal ovarian epithelial tissues (Figure 2(d,e)). In addition, immunohistochemistry of the tissue microarray HOvaC160Su01 illustrated the significant overexpression of WNK2 in the OC tissues (p < 0.001) (Figure 2(g) and Table 2). In this study, we found that WNK2 expression was the opposite of miR-324-3p in OC.

**Figure 2.** WNK2 is upregulated in ovarian cancer and indicates poor survival of OC patients. (a) Relative mRNA expression of WNK2 in normal ovarian epithelial cell IOSE-80 and three OC cell lines A2780, CAOV3, and SKOV3. (b) The protein expression of WNK2 in IOSE-80, A2780, CAOV3, and SKOV3. (c) Immunofluorescence staining of WNK2 in SKOV3 cell line. (d) WNK2 expression was analyzed in most normal tissues and cancer tissues in Human Atlas Protein Database. (e) TCGA database shows WNK2 were overexpressed in OC tissues. (f-g) Immunohistochemistry staining of WNK2 in OC and adjacent ovary tissues (***P < 0.001). (h) The expression of WNK2 in low and high-grade OC tissues (**P = 0.0068). (i) Upregulated WNK2 predicts poor survival of ovarian serous adenocarcinoma patients.

**Table 2.** WNK2 was increased in ovarian cancer and positively correlated with tumor pathological grade p < 0.05

Parameters	Total (n = 159)		P-value
	High WNK2 expression (119)	Low WNK2 expression (40)	
			Pathology types
Boderline tumors	1	4	0.038*
Serous carcinoma	80	16	
Mucinous carcinoma	19	14	
Other pathology types	19	6	
			Ages (years)
≧55	69	28	0.244
<55	50	12	
			TNM stage
I+ II	50	12	0.448
III+IV	88	35	
			pathology manignity
low grade	29	20	0.0068*
high grade	88	22	

### 3.4 WNK2 overexpression indicates the poor survival of patients with OC

Immunohistochemistry revealed the positive correlation between WNK2 expression and tumor pathological grade. The WNK2 levels in patients of different age groups and TNM stages were not significantly different. However, we observed a positive correlation between WNK2 levels and tumor malignancy (p < 0.05) (Figure 2(h)). Cox regression showed that in serous ovarian adenocarcinoma, the higher the WNK2 expression, the shorter the patients’ survival time (Figure 2(i)). These results suggest that WNK2 may promote OC proliferation and thereby malignancy.

### 3.5 WNK2 knockdown inhibits the proliferation and invasiveness of cancer cells

In WNK2-overexpressed OC cells (SKOV3 and CAOV3 cells), WNK2 was successfully knocked down at both the mRNA and protein levels (Figure 4(a)). Then, CCK-8, EdU, and colony assays were employed to evaluate the cells proliferation ability. Results illustrated that WNK2 knockdown significantly inhibited SKOV3 and CAOV3 cell proliferation (p < 0.05). Transwell assays indicated that WNK2 knockdown suppressed the invasiveness of the cancer cells (Figure 4(b–e)), and nude mouse models showed that tumors smaller than the control cells were formed when WNK2 was knocked down (Figure 4(f)). Immunohistochemistry (IHC) staining verified the efficiency of WNK2 knockdown in nude mouse tumors (Figure 4(g)).

**Figure 4.** WNK2 knockdown suppresses OC development both in vitro and in vivo. (a) Validation of WNK2 knockdown in SKOV3 and CAOV3 by western blot analysis and RT-qPCR. (b) With WNK2 knockdown, the proliferation of cell lines was analyzed by CCK-8 assay. (c) The invasiveness of cell lines was analyzed by Transwell assay. (d-e) Colony formation and EdU assays evaluated the viability of OC cells after WNK2 knockdown. (f) In vivo, WNK2 knockdown inhibited tumor growth. (g) Immunohistochemistry staining for WNK2 in nude mouse tumors. ** P < 0.01, *** P < 0.001.

### 3.6 WNK2 overexpression increased the proliferation and invasion of cancer cells

To further confirm the oncogenic role of WNK2, we transfected WNK2 plasmids into WNK2-under expressed A2780 and CAOV3 cells. Then, RT-qPCR and Western blotting verified the overexpression efficiency (Figure 5(a)). It was found that WNK2 overexpression increased the viability and invasive ability of A2780 and CAOV3 cells (Figure 5(b–e)). In general, WNK2 promotes OC progression.

**Figure 5.** WNK2 exerts tumor promoting roles in OC. (a) Validation of WNK2 overexpression in A2780 and CAOV3 by western blot analysis and RT-qPCR. (b) the viability of cell lines was analyzed by CCK-8 assay. (c) the invasion of cell lines was analyzed by Transwell assay. (d-e) Colony formation and EdU assays evaluated the viability of OC cells after WNK2 overexpression. ** P < 0.01, *** P < 0.001.

### 3.7 WNK2 activates the RAS pathway

The phosphorylation modification levels of most proteins decreased when WNK2 was knocked down. Kyoto Encyclopedia of Genes and Genomes (KEGG) enrichment analysis regards the RAS pathway as the most significant one (*P* < 0.01; Figure 6(a)). Moreover, we detected that the active GTP-bound conformatives (RAS-GTP) were reduced when WNK2 was knocked down (Figure 6(b)). These results indicated that WNK2 activates the RAS pathway.

**Figure 6.** miR-324-3p inhibits OC development by targeting WNK2/RAS pathway. (a) KEGG enrichment analysis of phosphorylation modification proteome profiling. (b) WNK2 knockdown reduced the level of RAS-GTP. (c) WNK2 partly reversed the viability suppression of miR-324-3p on OC cells. (d) WNK2 knockdown partly reversed the tumor promoting roles of miR-324-3p inhibitors on OC cells. ** P < 0.01, *** P < 0.001.

### 3.8 WNK2 reverses the effects of miR-324-3p on OC cells

Rescue experiments were performed to further confirm that WNK2 is a target of miR-324-3p. Figure 6(c,d) shows that WNK2 reverses the inhibitory effect of miR-324-3p on OC cells. Conversely, WNK2 knockdown weakened the miR-324-3p proliferation inhibitor (Figure 6(d)). In conclusion, *WNK2* is the target gene of the tumor suppressor miR-324-3p.

## 4. Discussion

Owing to the lack of sensitive diagnostic methods and effective therapies, OC has the highest death rate among gynecological cancer types. In recent years, miRNAs have attracted considerable attention as cancer diagnostic and therapeutic tools, and some of them have brought significant progression in clinical trials [38,39]. We have observed OC progression is inseparable from dysregulated miRNAs. For example, the well-known downregulated let-7 family plays tumor-suppressive roles in OC by targeting oncogenes, such as *c-MYC, HRAS*, and *KRAS*, and cell cycle regulators [40,41]. The miRNA-200 family, miR-506, and miR-122 are widely known to influence OC progression by modulating epithelial–mesenchymal transition (EMT) transcription factors [42]. Our study confirmed that miR-324-3p expression is decreased in OC, and inhibited the malignant proliferation of OC cells. miR-324-3p has the potential to be used as the diagnostic and therapeutic targets for OC [43].

miR-324-3p influences the phenotypes of various cancer cells by binding to critical targets. It can reverse the chemotherapy resistance of colon, nasopharyngeal, and lung cancer cells by targeting Wnt/β-catenin, *SMAD7* (SMAD family member 7), and *GPX4* (glutathione peroxidase 4) [13–18], and also regulates the progression of breast and pancreatic cancers by regulating ferroptosis and angiogenesis, respectively [15,44]. In breast cancer, its antitumor role is mediated by targeting of the SET domain-containing protein 1A (*SETD1A*)-PI3K-AKT pathway [18]. Bioinformatics websites predicted miR-324-3p to target the 3'UTR of *WNK2*, which was confirmed by luciferase assays in this study. Our study is the first to prove that miR-324-3p suppresses *WNK2* expression at both mRNA and protein levels.

WNK2 is a cytoplasmic protein with several domains. It plays critical roles in various cancers such as gliomas and gastric, breast, cervical, colon cancers [28–31]. For instance, WNK2 suppresses cervical cancer by negatively modulating the MEK1/ERK1/2 pathway [32]. In this study, we demonstrated the tumor-promoting role of WNK2 in OC and found that the expression of WNK2 was exactly the opposite of that of miR-324-3p in OC cells and tissues. And WNK2 expression is positively correlated with tumor malignancy and negatively correlated with patient prognosis, which not only facilitates OC progression both in vitro and in vivo but also reverses the cancer-suppressive effects of miR-324-3p. In summary, our study is the first to demonstrate that miR-324-3p inhibits the OC malignant behavior by targeting WNK2. Moreover, protein phosphorylation sequencing and experiments have illustrated that WNK2 activates the RAS pathway. As is well known, the abnormal activation of the RAS signaling pathway is the most common change in tumors [45,46]. RAS signaling are indispensable for cancer pathogenesis [44]. In addition, sufficient evidence is available to prove that the occurrences of tumors are caused by RAS mutations and by the deregulation of downstream effectors. For instance, PI3K/AKT and MERK/ERK are vital effector pathways of Ras signaling, contributing to OC proliferation and migration [47–49]. The upstream and downstream of the RAS pathway may be considered as potential cancer therapeutic targets [50,51]. Our research suggests that *WNK2* is a target of miR-324-3p, and miR-324-3p suppresses OC proliferation by targeting the WNK2/RAS pathway. In summary, we have provided a theoretical basis for miR-324-3p to act as an OC diagnostic and therapeutic tool. However, we haven’t revealed how WNK2 activates Ras pathway. In a future study, we will try to elucidate the mechanism, and treat OC by introducing miR-324-3p mimics or miR-324-3p delivery systems, such as DNA plasmids or small molecules, into cancer cells.

## 5. Conclusion

In summary, this study revealed that miR-324-3p inhibited OC development by targeting the *WNK2*/RAS pathway. Moreover, the OC cancer-promoting role of WNK2 has also been demonstrated. We hope that both miR-324-3p and WNK2 can be used as diagnostic markers and potential therapeutic targets for OC treatment.
